# A Few-Shot Learning-Based Siamese Capsule Network for Intrusion Detection with Imbalanced Training Data

**DOI:** 10.1155/2021/7126913

**Published:** 2021-09-13

**Authors:** Zu-Min Wang, Ji-Yu Tian, Jing Qin, Hui Fang, Li-Ming Chen

**Affiliations:** ^1^College of Information Engineering, Dalian University, Dalian 116622, China; ^2^School of Software Engineering, Dalian University, Dalian 116622, China; ^3^Department of Computer Science, Loughborough University, Loughborough LE113TU, UK; ^4^School of Computing, Ulster University, Belfast NIC100166, UK

## Abstract

Network intrusion detection remains one of the major challenges in cybersecurity. In recent years, many machine-learning-based methods have been designed to capture the dynamic and complex intrusion patterns to improve the performance of intrusion detection systems. However, two issues, including imbalanced training data and new unknown attacks, still hinder the development of a reliable network intrusion detection system. In this paper, we propose a novel few-shot learning-based Siamese capsule network to tackle the scarcity of abnormal network traffic training data and enhance the detection of unknown attacks. In specific, the well-designed deep learning network excels at capturing dynamic relationships across traffic features. In addition, an unsupervised subtype sampling scheme is seamlessly integrated with the Siamese network to improve the detection of network intrusion attacks under the circumstance of imbalanced training data. Experimental results have demonstrated that the metric learning framework is more suitable to extract subtle and distinctive features to identify both known and unknown attacks after the sampling scheme compared to other supervised learning methods. Compared to the state-of-the-art methods, our proposed method achieves superior performance to effectively detect both types of attacks.

## 1. Introduction

Network intrusion detection systems (NIDS) play important roles in network security in the past several decades [1–3]. NIDS can distinguish abnormal network attacks from routine network traffic, thus ensuring communications safety. Many deep-learning-based methods, including deep autoencoder [4], convolutional neural network [5], and LSTM [6], have been proposed in recent NIDS studies to identify various complex, unknown attacks resulted from the growing popularity of the Internet of Things and cloud-based services [7]. Compared to the traditional machine learning methods, such as SVM [8], KNN [9], random forest [10], and boosting [11], deep-learning-based algorithms, have demonstrated better performance to address the growing complexity and diversity of types of attack.

Despite substantial advances being made, there exist two major challenges in designing a reliable and effective NIDS, namely the imbalanced training data sets and the frequent occurrences of unknown attacks. In information systems, normal samples in network traffic are sufficient, easy to obtain, and diverse in subtypes. However, it is very difficult to obtain network attack samples because abnormal flow accounts for a small proportion of total flow, and traffic samples of newly emerging forms of attacks such as “zero-day” attacks are difficult to obtain.

To address the imbalanced data problem, either over- or undersampling strategy has been proposed to balance the training data [12–14]. However, each strategy has its own weakness in practice. The oversampling scheme, as mentioned in [15], is difficult to find an appropriate distribution to oversample the abnormal intrusion attacks, whereas the undersampling strategy generates less data that may cause overfitting issues for training an effective classifier. In addition, most advanced deep-learning-based NIDS classifiers are less sensitive to unknown attacks as they are trained by maximizing the possibility that a sample belongs to one known attack type. A classifier's performance is highly dependent on the traffic characteristics used in the training process, so it is difficult to identify unknown attacks in the detection process, thus unable to cope with the changing network environment.

To address the above-mentioned challenges, in this paper, we propose a novel NIDS algorithm that integrates an unsupervised subtype sampling scheme with a few-shot learning-based Siamese capsule network to achieve reliable detection of different types of network attacks as well as identify new unknown attacks effectively. Specifically, we design a new sampling method based on unsupervised machine learning techniques, for example, clustering to group training samples of each network attack type into subtypes of data. With this method, more representative samples can be preserved when balancing the training data. These samples are then used to train the few-shot learning-based Siamese capsule network so that subtle patterns and distinctive features can be extracted by a metric learning framework. These two components are complementary to build a reliable and effective NIDS.

Recently, there are several few-shot learning-based intrusion detection methods proposed in [16–18]. These methods can build an effective detection model with only a small number of samples, and the similarity measurement mechanism in methods is very suitable for dealing with unknown attacks. Compared to previous studies, the distinctive advantages of the new data-processing method and the improved algorithm structure have made the proposed method outperform them. Overall, the contributions of our method are highlighted as follows:

- We propose a new unsupervised subtype sampling mechanism to construct a few-shot learning training data set with an indefinite *K* value from an unbalanced data set. This scheme can obtain large representative samples by clustering the training data of each attack type into subtypes, thus taking data distribution into consideration. It further improves the reliability of the few-shot learning network performance.
- We develop an innovative Siamese capsule network by adapting the capsule network architecture into the Siamese network for intrusion detection. As a result, the location information across features can provide extra cues to help detect distinctive patterns of intrusion attacks.
- We redefine a so-called *C*-way *K*-shot *E*-extra problem in the context of a few-shot learning framework in the field of intrusion detection so that our approach can detect unknown attack types without samples. When facing unknown attacks, this is more like a special zero-shot learning method based on few-shot learning [19]. In the experiment, we found that the support set and the similarity comparison method are the main factors affecting the detection accuracy of unknown types.

The remainder of this paper is organized as follows.  Section 2 discusses related works to provide the background of our approach.  Section 3 explains the proposed NIDS methods in detail.  Section 4 presents experimental results to demonstrate the effectiveness of our method and its performance comparing to the state-of-the-art methods. Finally, Section 5 concludes the paper and identifies future work.

## 2. Related Works

In this section, several issues in NIDS that are relevant to this paper are discussed separately, including network intrusion detection techniques, method of unbalanced data processing, and few-shot learning. A compilation of related work is shown in Table 1.

### 2.1. Network Intrusion Detection Techniques

Network intrusion detection systems are usually used to detect various malicious traffic in information systems. Thus, they can be defined as binary classification systems to distinguish between normal and malicious network traffic. Wang et al. [8] proposed an intrusion detection framework based on a support vector machine (SVM). This method applies the logarithm marginal density ratios transformation to form original features with the goal of obtaining new and better-quality transformed features that can improve the detection capability of an SVM-based detection model. As an excellent classifier in machine learning, the XGBoost algorithm is also applied in the field of intrusion detection. The detection model proposed by Su et al. [11] relies on XGBoost to obtain high detection accuracy. A fuzzy rule-based automatic intrusion detection system [20] is proposed as a solution to deal with precise measurement and uncertainty in the judgment of each criterion. Furthermore, fuzzy TOPSIS (Technique for Order of Preference by Similarity to Ideal Solution) is used for response prioritization in multicriteria decision-making. Iannucci and Abdelwahed [21] proposed a probabilistic model-based intrusion detection system built on a multiagent discrete-time Markov decision process (MA-MDP), which effectively captures the dynamics of both the defended system and the attacker. This model is used to automatically compose response actions to plan a multiobjective long-term response policy in order to protect the system.

Recently, deep learning-based algorithms are widely used in intrusion detection due to their excellent performance in classification tasks. Wu et al. [22] proposed an intrusion detection method using a convolutional neural network. This method converts the vector format of the original data into an image format. Consequently, the CNN algorithm is used to extract traffic characteristics and builds an intrusion detection model through training. The method proposed by Mirza and Cosan [6] exploited an autoencoder to project sample data into a latent space, extract features through the LSTM algorithm, and then determine whether an incoming network data sequence is abnormal through a preestablished threshold. Compared with LSTM, GRU neural network is more suitable for real-time processing. Thus, Yan and Han [23] utilized the time relationships between network traffic and used GRU as a classifier to detect abnormal traffic. Furthermore, both Wang et al. [24] and Vinayakumar et al. [5] demonstrated that combining CNNs and RNNs to extract the temporal and spatial characteristics of network traffic could achieve great performance of classifying normal and abnormal traffic. Since the efficiency and accuracy of the NIDS method of detection are equally important, Mirsky et al. [25] proposed a method based on the integration of artificial neural networks and self-encoders (Kitsune) for unsupervised anomaly detection tasks. The detection performance of this method can be gradually improved over time. Bovenzi et al. [26] further proposed a lightweight solution based on multimodal deep autoencoder (M2-DAE), which supports distributed deployment and is able to manage numerical and categorical features efficiently.

### 2.2. Method of Unbalanced Data Processing

To address the imbalanced training data problem, extensive research has been undertaken in preprocessing training data [27–29] as the extreme imbalanced data sets between various types of traffic attacks have greatly limited detection performance.

Yilmaz et al. [30] proposed to generate samples of various attack types through the GAN network to construct a balanced training data set. Caminero et al. [31] embedded GAN into a classifier and extracted samples from the data set based on reinforcement learning to generate new samples and adjust this initial sample generation behaviour through an adversarial network. However, it is still a challenge to simulate data samples with unknown data distributions with the convergence of GAN models. The method proposed by Zhang et al. [14] used SMOTE oversampling and GMM clustering algorithm for under- and resampling all types of samples to achieve uniformity. Similarly, Engly et al. [32] created an imbalance-corrected data set using SMOTE's algorithm and then used three different methods for feature selection on the data, such as correlation-based, fast correlation-based, and consistency-based methods. Lopez-Martin et al. [33] used the generative model of a variable autoencoder (VAE) in their work. Their model generated samples based on the distribution of labels. Compared to other oversampling methods, the process of this method is simpler, more reliable, and faster. Yang et al. [34] proposed an improved density peak clustering algorithm (MDPCA) data preprocessing method to divide large-scale network data into several training subsets of different clustering centres. This method breaks the imbalance of multiple types of data and achieves feature dimensionality reduction. Wang et al. [35] proposed a novel probabilistic detection framework of weighted combining semisupervised *k*-means clustering and posterior probability SVM (PPSVM) for unbalanced data based on robot vision and achieved a relatively significant improvement in detection performance. While significant progress has been made, challenges remain for these existing preprocessing methods. For example, synthesizing samples using oversampling techniques can reduce the sample quantity gap between classes but increase the likelihood of overlapping samples within classes, thus creating samples that do not provide valid information. Undersampling balances the number of samples between types by reducing the number of sufficient classes but is prone to overfitting. In a nutshell, data augmentation alleviates overfitting in low data regimes but does not solve it.

### 2.3. Few-Shot Learning

To address the detection of unknown attacks, few-shot learning models have been proposed to solve tasks with a limited number of training samples [36]. The models mainly include prototypical networks [37], relational networks [38], matching networks [39], and Siamese networks [40]. Among them, the prototype network [37] provides the support set and the query set so that it turns the classification problem into the nearest neighbour problem in the embedding space. In contrast, the matching network [39] uses two different embedding functions for the support set and the query set. The output of the classifier is a weighted sum of the predicted values between the support set samples and the query set. The relationship network [38] calculates the distance between two samples by constructing a neural network to analyze the degree of matching. The Siamese network [40] constructs a parallel neural network with shared weights. During training, sample pairs are constructed by random combination as the input of the Siamese structure, and the distance between the sample pairs is calculated to measure the similarity between the sample pairs. During the test, the Siamese network takes pairs of the tested sample and the different types of samples in the support set as input and treats the sample type with the highest similarity between the support set and the tested sample as the type of the tested sample.

Recently, two few-shot learning methods for intrusion detection have been proposed by Yu and Bian [17] and Xu et al. [18]. The former exploits a deep convolutional neural network algorithm that is integrated into the metric learning network to calculate the Euclidean distances of different samples to further distinguish between normal traffic samples and attack traffic samples, whereas the latter [18] further processes traffic data from spatial and temporal features. The method combines temporally adjacent samples in the same connection into spatial three-channel images and uses Conv3D's convolution operation to construct a Siamese network to detect image-based intrusion events. Obviously, the deep learning algorithm still occupies a vital part of the few-shot learning method. In contrast, the Siamese networks model in the latter [18] is more scalable and can be embedded with different algorithms to extract the underlying features of the traffic data. However, this method ignores the global spatial distance between classes, which is not conducive to the improvement of detection accuracy.

## 3. The Proposed Approach

The architecture of our proposed approach is illustrated in Figure 1. Central to the approach is the notion of two Siamese capsule networks that provide a parallel network structure to achieve directed feature extraction from different traffic samples. The general idea is that in the training phase, the network relies on a small number of samples to obtain an effective detection model without falling into overfitting. Then, in the testing phase, the similarity comparison method can be used to effectively classify abnormal samples that are not included in the training set. As the few-shot learning structure is robust in addressing sample scarcity and imbalance in the learning process, the proposed approach offers a promising solution for intrusion detection including unknown sample types.

Specifically, the approach will work as follows. At the training stage of our intrusion detection algorithm, data samples from different types of attacks and normal network traffic are clustered and sampled based on the proposed unsupervised subtype sampling scheme, which is explained in the next subsection. After resampling the raw data set, the balanced data set and data samples collected from scarce attack types are used to form the training set for the Siamese capsule network training so that the few-shot learning algorithm could learn more distinctive features to identify the network attacks with such imbalanced data set. In addition, the balanced few-shot training set is used as the support set at the test stage to identify the abnormal network behaviours. At the test stage, we use the most similar samples in the support set to classify the tested samples after extracting features from the Siamese capsule network. It is to be noted that two-dimensional grayscale images converted from the traffic vectors are built as the input feature representations of the proposed framework. The detail of the representation is explained in the experiment in Section 4.1.

### 3.1. Unsupervised Subtype Sample

#### 3.1.1. Unbalanced Data Set

Learning tasks in scenarios with unbalanced sample numbers have received extensive research attention. Although a large volume of normal traffic data could be easily collected, training samples of intrusion attacks are usually much scarcer. When dealing with unbalanced data sets, traditional methods usually use data enhancement and enrich supervision information to construct new balanced data sets [41]. The specific operation is to repeatedly undersample the types with sufficient samples and discard some redundant samples. For the types with scarce samples, new samples are generated by algorithms such as GAN to balance the number of samples in the sufficient and scarce classes [42]. However, simulating data samples from arbitrary data distributions using GAN is still a challenging task. Similarly, cost-sensitive learning can deal with the sample imbalance between classes. However, the method still needs to rely on large-scale samples and is not the key to solve the sample scarcity problem. Furthermore, cost-sensitive learning pursues classification cost more than classification accuracy, which is not feasible for many detection tasks [43]. In contrast, few-shot learning is built on top of the metric learning structure, which can better capture unknown attacks.

The “*C*-way *K*-shot” in few-shot learning is a learning method, which constructs *C* categories, and each category has *K* samples. In this method, the value of *K* for each category is usually fixed and identical. However, the intra- and interclass variations of traffic data in network intrusion detection vary when the *K* value is changed. If the value of *K* is much smaller than the type of its subtype, the learning ability of the algorithm for normal samples will be insufficient, which will affect the detection performance. On the contrary, if a high *K* value is set, the subtypes may have too few samples as the sample number of newly emerging attacks is sparse. Therefore, it is still difficult to build a suitable few-shot training set using a fixed *K* value. In our method, instead of pursuing the balance between samples and categories, we set the *K* value as an adaptive value, that is, the value of *K* is different in different types. In this way, we are able to fully learn the features in normal types, while avoiding the restriction on *K* values of sparse classes.

To illustrate the variations of traffic samples of different types of attacks, we randomly sample six types of attacks, including Benign, Bot, DDoS, PortScan, DoS GoldenEye, and Web Attack SQL Injection in the CICIDS-2017 data set [44] and randomly select two different features to display the data distributions. As shown in Figures 2(b), 2(c), 2(f), and 2(i), Bot-type samples are distributed loosely across the feature spaces of Avg Fwd Segment Size, Packet length Variance, Packet Length Std, Fwd Packet Length Mean, and Subflow Fwd Bytes. In contrast, there are distinctive differences between samples in the same attack types. As illustrated in Figures 2(a), 2(d), 2(e), 2(h), and 2(i), samples in some attack types, for example, the types such as Benign and DoS GoldenEye with respect to the features Fwd IAT Mean and Active Max, are densely distributed, and they could be clustered well.

In an information system, the normal traffic of the HTTP protocol and the SNMP protocol behave differently in connection characteristics, traffic characteristics, and header content; even the normal traffic within the HTTP protocol is different. As the goal of traffic attacks is to disguise normal samples from all levels, many samples of the attack data have significant variations in characteristics, while samples of different attack types share similarity in some characteristics. Therefore, when constructing a few-shot data set, it is required to design a sampling scheme to obtain sufficient samples to cover each subtype of these attacks.

#### 3.1.2. Unsupervised Subtype Sampling Method

As shown in Figure 3, when performing unsupervised subtype sampling, first, we use an adaptive *k*-means method [45] to cluster the samples into subtypes of each attack type for our resampling scheme. Each subtype is then randomly sampled one by one to obtain a subset representing that type available for training. The *K* number is determined adaptively based on the silhouette coefficient [46], which balances cohesion and separation factors as shown in the following equation:

(1) $$\begin{array}{c} S\left(i\right)=\frac{b\left(i\right)-a\left(i\right)}{\max\left\{a\left(i\right)-b\left(i\right)\right\}}, \end{array}$$

where *a*(*i*) represents the average of the distances from the samples *i* in the cluster to all other samples in the cluster and *b*(*i*) represents the minimum value of the average distance from the sample *i* in the cluster to all samples in the cluster closest to the sample. The calculation result of the silhouette coefficient is between −1 and 1. After setting a set of candidate *K* values and run the *k*-mean method to cluster the data in each attack type, the final *K* value for each type is selected based on the following equation, which is the smallest number of clusters from the top *n* largest silhouette coefficient.

(2) $$\begin{array}{c} K=\min\left\{\arg\max_{n}\left\{S\left(2\right),S\left(3\right),\ldots ,S\left(i\right)\right\}\right\}, \end{array}$$

where the parameter *n* is usually set to 10 and argmax_*n*_ represents the number of clusters corresponding to the largest first *n* silhouette coefficient. After obtaining the most appropriate number of clusters, we take one sample from each subtype after clustering to build a few-shot training set of sufficient classes. In contrast, this new sampling method is able to select representative samples from sufficient classes for training and can alleviate the problem of information loss in random undersampling. As shown in Figure 2, after unsupervised clustering is used to obtain a type of set with subtype labels, a sample is drawn from different subtypes, and a subset of this type is generated as a training set.

We illustrate the sampling results in Figure 4. Here, 1,000 samples without labels were randomly selected on the normal traffic type, and the *K*-means algorithm was used for clustering. According to the above unsupervised subtype sampling method, the optimal number of clusters is 20. After completing the clustering, a sample is randomly selected from each subtype to observe the distribution of unsupervised sampling samples in all samples. As shown in Figure 4, a small set consisting of 20 samples is evenly distributed on different features, with a high degree of dispersion, and has a high representative value for each feature.

### 3.2. The Directed Few-Shot Network-Based NIDS

#### 3.2.1. Siamese Network

Siamese network is an application form of few-shot learning in the field of supervised learning framework. Its main goal is to learn a reliable classification model based on a very small number of samples. It is also considered as one type of metric learning method, which classifies samples by comparing the similarity between the tested samples and the labelled samples in its support set. The classification task establishment process is as follows:

  Step 1: determine the number of types *C* and the sampling value *K* of each type. Construct a few-shot learning data set, including training set, query set, support set, and test set.
  Step 2: choose suitable feature extraction neural network algorithms to construct a backbone network with weight sharing and choose a suitable similarity measurement method to construct a comparison network.
  Step 3: randomly sample the same type and different types of sample pairs as the input of the Siamese network. If the two samples in the input sample pair are of the same type, the similarity label is 1, and if the types are different, the similarity label is 0.
  Step 4: compare the output label with the real label to obtain the loss and establish the network model step by step iteratively.
  Step 5: bring the sample pair composed of the tested sample and the sample in the support set into the model to measure the similarity. Take the sample type in the support set with the highest similarity to the tested sample as the tested sample type.

#### 3.2.2. The CapsuleNet Method

The main function of the Siamese backbone network is to extract features from samples. CNN can effectively extract features, but it also has certain limitations. First, the data is transferred between neurons in a scalar way. Scalar has only content but no direction, so CNN is not strong in recognizing the spatial position relationship between features. Second, the pooling layer of CNN will lose a lot of valuable information. The characteristic location of the network traffic sample is very sensitive [47], and the confusion of the location relationship will inevitably affect the accuracy of the judgment result. The capsule network transmits information in the form of vectors, which can effectively characterize the location and direction of features. In addition, the dynamic routing algorithm of the capsule network avoids the feature loss caused by the pooling operation. Thus, there are two main motivations for us to use the capsule-based architecture in our work: firstly, a network intrusion attack typically generates very salient local features. Compared to other deep learning architectures, capsule-based network architecture has a distinctive advantage of using a local feature for classification, which naturally fits the NIDS task. Secondly, classical convolutional neural network architectures use the max-pooling operation to explore the relationship between features. While this operation causes information loss in higher-level features extracted from the networks. In contrast, the capsule-based network architecture utilizes dynamic routing to replace the max-pooling operation. Considering that the feature space of NIDS is relatively small that cannot afford the information loss caused by the max-pooling operation, it is believed that the capsule-based network architecture is more suitable for NIDS. We develop the CapsuleNet method as the backbone of our Siamese backbone network, as illustrated in Figure 5.

Although the capsule network guarantees the directionality of the feature extraction process, the initial process of extracting features from the original data still needs to rely on the convolution operation. As shown in Figure 5, after a sample is feature extracted through the initial convolution operation, the feature is converted into a vector through the Primary Caps layer as the input of the dynamic routing algorithm. The dynamic routing algorithm outputs a feature vector representing image features after a series of operations such as matrix transformation, input weighting, summation, and nonlinear transformation are performed on the vector. The output of the final capsule network can be used as the input of the comparison network. Due to space limitations, the specific calculation process of the dynamic routing algorithm between capsules can be found in the literature [48].

#### 3.2.3. Using Siamese Capsule Network for Intrusion Detection

In our work, we propose the Siamese capsule network for the NID system. As the metric model is a crucial part of the few-shot learning method, the Siamese network is used in our work. As illustrated in Figure 6, the Siamese-directed network constructed by combining few-shot learning, and capsule network can effectively deal with the problem of scarce attack samples and sensitive sample feature positions in intrusion detection.

As shown in Figure 6, in the backbone network with shared weights, the sample obtains the feature vector after initial feature extraction through a two-dimensional convolution operation. After the features are reshaped, they are input into the capsule network for directional extraction, and Flatten is used to compress the vector output from the capsule network in one dimension. The one-dimensional vectors of different samples are compared for similarity in the comparison network. First, these two one-dimensional vectors are subtracted, and then the absolute value is added. It is equivalent to obtaining the norm of the difference between the two eigenvectors. Then, it is fully connected to this norm twice, and the second time, it is fully connected to a neuron. Finally, the Sigmoid activation function is used to activate the output of this neuron, so that its value is between [0, 1], which represents the degree of similarity between the two input pictures. Although the Siamese network using random sample pairs can achieve multiclassification tasks, in fact, according to the input of the Siamese network, the training task is still carried out according to the binary classification. Therefore, we use binary cross-entropy to calculate the loss [49]; the formula is as follows:

(3) $$\begin{array}{c} L\left(x_{1}^{i},\;x_{2}^{i}\right)=y\left(x_{1}^{i},\;x_{2}^{i}\right)\log\;p\left(x_{1}^{i},\;x_{2}^{i}\right)+\;\\ \left(1-\;y\left(x_{1}^{i},\;x_{2}^{i}\right)\right)\log\;\left(1-p\left(x_{1}^{i},\;x_{2}^{i}\right)\right)+\lambda T\;|w, \end{array}$$

where *x*_1_^*i*^, *x*_2_^*i*^ are two random samples input at one time. If the samples are of the same type, *y* (*x*_1_^*i*^, *x*_2_^*i*^) = 1, otherwise, it is *y* (*x*_1_^*i*^, *x*_2_^*i*^) = 0. In addition, we also use the Adam optimizer with better convergence performance [50]. To solve the problem of insufficient generalization ability, the decay mechanism is introduced to update the learning rate with the epoch. The pseudocode of generating the training set and the proposed network training are provided as Algorithms 1 and 2.

## 4. Experiment

### 4.1. Experimental Data and Environments

To evaluate the detection effect of the proposed methods, we conduct experiments using the CICIDS-2017 data set [44] and UNSW_NB15 data set [51]. CICIDS-2017 contains 14 attack samples and 1 normal sample. According to the definition of few-shot learning, 8 sample types are selected, including normal type and 7 attack types. UNSW_NB15 contains 9 attack samples and 1 normal sample. According to the definition of few-shot learning, 7 sample types are selected, including 1 normal type and 6 attack types. To simulate the imbalance of data, three types, namely sufficient, scarce, and zero-sample, are categorized. The specific distribution is shown in Table 2.

Among the selected 7 attack types on the CICIDS-2017 data set, we define 5 of them as known attack types. The other 2 attack forms (iG and iH) simulate unknown attacks, and there are no samples of these two types to be used in the training set. Among the known attack types, the iB and iC attack types are set to have sufficient traffic samples, and the iD, iE, and iF attack types have limited traffic samples. Each sample in the data set has 78 features and 1 sample label. We set *N* = 9 and establish each sample as a 9 ∗ 9 grayscale image to extract geometric features.

Among the selected 6 attack types on the UNSW_NB15 data set, we define 4 of them as known attack types. The other 2 attack forms (rF and rG) simulate unknown attacks, and there are no samples of these two types to be used in the training set. Among the known attack types, the rB and rC attack types are set to have sufficient traffic samples, and the iD and rE types have limited traffic samples. Each sample in the data set has 49 features and 1 sample label. We set *N* = 7 and establish each sample as a 7 ∗ 7 grayscale image to extract geometric features.

#### 4.1.1. Training Set

We conduct experiments under two different settings to simulate the imbalance of data in practical applications. CICIDS-2017 data set is taken as an example, in the first setting; we set the maximum number of training samples for the Benign, DDoS, and Bot types in abnormal traffic to 1,500, 1,000, and 500, respectively, and the maximum number of training samples for scarce attack types PortScan, DoS GoldenEye, and Web Attack SQL Injection to 5, 5, and 5, respectively. In the second setting, we set the maximum number of training samples for the Benign, DDoS, and Bot types in abnormal traffic to 3,000, 2,000, and 1,000, respectively, and the maximum number of training samples for scarce attack types PortScan, DoS GoldenEye, and Web Attack SQL Injection to 20, 20, and 10, respectively. After obtaining different types of available training data sets, value samples are selected to form the training data set through unsupervised subtype sampling and establish multiple training sets with different sample sizes to verify the usability of the method. The UNSW_NB15 data set is the same in the selection strategy of the training set. As shown in Table 3, training A and training B denote two training sets with different sample sizes.

#### 4.1.2. Implementation and Experiment Environments

The experiment was carried out under the environment of CPU Intel Xeon E5-2620, GPU NVIDA GTX1080ti, RAM 64G, video memory 11G, CuDNN 7.6.5, CUDA 11.0, TensorFlow 1.13.1, and Keras 2.2.4.

### 4.2. Evaluation Metrics

In addition, to test the classification on the known attacks, the detection task is also tested on unknown attacks. The classification of unknown attack samples relies on the comparison of their similarity with normal samples and abnormal samples. Therefore, the model's detection of traffic samples is a process of binary classification of normal samples and abnormal samples. The test results of the samples are divided into the following four types:

1. TP: normal samples are correctly detected as normal samples
2. FN: normal samples are incorrectly classified as abnormal samples
3. TN: attack samples are correctly detected as abnormal samples
4. FP: attack samples are incorrectly classified as normal samples

We use three evaluation indicators including accuracy rate, precision rate, and recall rate to evaluate the method. The accuracy rate is the ratio of the number of samples correctly classified to the total number of samples, which can reflect the accuracy of the model classification. The precision rate is the proportion of real positive samples in the samples that are judged to be positive. The recall rate refers to the proportion of samples that are judged to be positive in all samples that are truly positive. The latter two items can reflect the classification performance of the method from two aspects: false positives and underreports. The formulas of each evaluation standard are as follows:

(4) $$\begin{array}{c} \text{accuracy}=\frac{\left(\text{TP}+\text{TN}\right)}{\left(\text{TP}+\text{TN}+\text{FP}+\text{FN}\right)},\\ \text{precision}=\frac{\text{TP}}{\left(\text{TP}+\text{FP}\right)},\\ \text{recall}=\frac{\text{TP}}{\left(\text{TP}+\text{FN}\right)}. \end{array}$$

The above three evaluation criteria can effectively judge the detection accuracy of the method, but in order to better show the model's ability to detect attack traffic, we introduce the detection rate to further evaluate the method. The detection rate refers to the proportion of samples that are correctly judged as negative classes in the entire negative class samples, that is, the proportion of detected attack samples occupying all attack samples. The expression formula is as follows:

(5) $$\begin{array}{c} \text{detection rate}=\frac{\text{TN}}{\left(\text{TN}+\text{FP}\right)}. \end{array}$$

### 4.3. Validation of Effects of Different Parameters and Backbone Structures

The Adam optimizer can maintain fast convergence but has insufficient generalization ability. After being supported by the decay strategy, its loss function converges more smoothly. As shown in Figure 7, when epoch = 500, the loss tends to stabilize, and the loss value decreases from 0.7 to 0.0006. Therefore, in the following experiment, the epoch is set to 500.

To verify the superiority of our proposed method, we also compare our method with different backbone networks that are integrated into the Siamese network. The DCNN network proposed by Yu and Bian [17], the VGG16 network proposed by Simonyan and Zisserman [52], and the ResNet18 network proposed by He et al. [53] are typical CNN algorithms that have achieved relatively successful applications in few-shot learning scenarios [54]. Thus, they are selected to compare with the proposed Siamese capsule network on the known attack test set. The performance of different algorithms on accuracy, precision, and recall is shown in Figure 8.

On training A of CICIDS-2017, the few-shot capsule network demonstrated an overall advantage with accuracy and recall of 98.37% and 96.29%, respectively. While ensuring a high accuracy rate for all samples, the Siamese capsule network algorithm can achieve an 86.55% abnormal detection rate, which is relatively stable performance. On training B, compared with the other two Siamese network algorithms, the Siamese capsule network still maintains a leading advantage as a whole. Although its detection rate of anomalies is slightly lower than that of the capsule network algorithm, it maintains a leading position in comprehensive evaluation criteria such as accuracy and recall. The experiments on the UNSW_NB15 data set further demonstrate the superiority of the method in the paper, maintaining the lead in the correct classification of both abnormal samples and normal samples. According to Figures 8(a)–8(d), it can be seen that with the increase of samples, the detection results are more stable. After multiple rounds of random experiments, from the perspective of various evaluation criteria, compared with other algorithms, the few-shot capsule network can achieve stable and accurate detection.

### 4.4. Results and Comparisons

#### 4.4.1. Validation of Unsupervised Subtype Sample Method

To test the sampling effect of the unsupervised subtype sample method, resampling method [17], random sampling [18], and sequential sampling without any sampling method are used for comparison on the data set mentioned in Section 3.1. According to the principle of the ablation experiment, the sampling method is set as the only variable, and other variables are kept uniform and fixed according to the proposed parameters in Table 3. Sequential sampling is to sample each type according to the order of the samples on the data set available for training. It is foreseeable that the samples obtained by sequential sampling must not have too much discreteness. Random sampling is to construct a data set by randomly drawing samples from different types. Resampling is divided into oversampling and undersampling. We use random sampling on types of sufficient to complete undersampling and use the GAN algorithm to oversampling to generate scarce classes samples to complete the construction of the resampled data set. Considering the randomness of the sampling process of various sampling methods, we conduct 10 experiments on various sampling methods respectively. The performance of the sampling methods on the test set is as follows.

As shown in Figure 9, the optimal detection results of different sampling methods are selected for comparison. The random sampling (RaS) method does not perform well in the application scenario where a small number of large-scale samples are sampled. Using resampling (ReS) to establish a balanced sample is better than random sampling, but there is still a big gap compared with an unsupervised subtype sample (US). In addition, from Figure 9(b), the detection result output by the unsupervised subtype sample method is more stable, which is a very important feature in the intrusion detection method. From the perspective of evaluation indicators such as accuracy and detection rate, the detection accuracy of the few-shot data set constructed by the unsupervised subtype sample method is much higher than that of the other three sampling methods, and it is more suitable for constructing a few-shot learning data set.

#### 4.4.2. Comparison of Few-Shot Learning Methods

To pursue higher detection accuracy, the method mentioned in [18] considers the time characteristics of the flow data when establishing the sample. The training set is divided into a sample set and a query set, which are constructed by random sampling according to the determined *K* value. The support set is established using a small amount of random sampling method. Its Siamese network architecture using FC-NET is constructed by a deep neural network (DNN). When testing, the tested sample is compared with the samples in different types of support set, and the type of the tested sample is judged by the size of the average value of each type in the tested sample support set. The difference between the above method and the method proposed in this paper is shown in Table 4.

To show the application effect of the method in the intrusion detection field, the few-shot learning method mentioned in the literature [18] is compared with the method mentioned in the paper on the test set containing known attacks and unknown attacks. The detection results of different methods on each evaluation index are shown in Table 5.  Table 6 shows the detection rates of various methods for different types of attacks.

In Table 6, on training A, there is no significant difference in the detection rate of different types of attacks by each method. However, combining the accuracy, precision, and recall rates in Table 5, the method in this article is higher in detection accuracy than the other two methods. Tables 5 and 6 shows that the detection rate of anomalies in the training set with the number of samples from small to large increases accordingly. On the B training set, the detection rate of the method in this article for iB and iE attack types is 100%, and the detection of rE attack types can also reach 99.5%. The comprehensive detection rate of various abnormalities can reach more than 90%, which exceeds the other two types of few-shot abnormality detection methods.

When facing unknown attack types such as iG, iH, rF, and rG, on the data set of *K* = 5, the FC-NET method has a better detection effect on unknown anomalies. However, as shown in Table 5, the accuracy of the FC-NET method can only reach 88.09% on the CICIDS-2017 data set and 88.65% on the UNSW_NB15, and its detection effect on unknown anomalies is at the expense of its accuracy. With the small increase in the number of samples, the detection rate of the detection method in this article for unknown attacks surpasses the other two methods, and the overall accuracy is higher. The detection rate of this method for unknown types of iG can reach 93.1%, surpassing FC-NET's 66.3%, and it also maintains a very high accuracy rate for normal types and known attack types.

#### 4.4.3. Comparison of Detection Results of Advanced Methods

In addition to comparing the above few-shot learning method recently proposed and applied in the field of intrusion detection with the method in the article under the same conditions, we also included other methods for comparison on different data sets. As shown in Table 7, compared to other methods, the method proposed in the article only uses a very small number of samples for training to achieve high detection accuracy. Moreover, the method proposed in the article also has the advantage of detection of unknown attacks. On training B, if the detection of unknown attacks is not included, the method can reach 96.26%, 99.07%, and 96.70% in accuracy, precision, and recall, respectively. Compared with the method using the same data sets [55, 56], the method in this paper has a better performance in detection accuracy. Even compared with other advanced methods that use a large number of samples for training [43, 53], the overall performance of this method is still not behind. However, compared with other methods of training on large-scale data sets through deep learning algorithms [57], this method is still slightly inadequate. But this does not conceal the value of this method, because the extremely low requirement on the number of samples and outstanding detection capabilities for unknown attacks are closer to intrusion detection in real scenarios. Furthermore, we compare the computational complexity of different algorithms by inference about floating points of operations (FLOPs). The efficiency of our proposed method is comparable to all advanced methods as a metric learning method based on a conjoined structure in addition to the highest accuracy performance we achieved. Moreover, compared with FC-NET, an advanced method achieving state-of-the-art performance mentioned in Section 4.4.2, our method has only 5% of the FLOPs of the former, which can be better adapted to the practical applications of intrusion detection.

## 5. Conclusions

In this paper, we designed a novel few-shot learning-based intrusion detection method with imbalanced training data. This method uses unsupervised subtype sampling to establish a few-shot data set with adaptive *K* values and builds a Siamese capsule network that can perform directed feature extraction. The experimental results show that we have achieved high accurate classification rate using only a very small number of samples, on the detection of both known attacks and unknown attacks. The detection of unknown attacks in our work is particularly outstanding due to the advantage of the metric learning framework.

In future research, we will further explore the temporal information to embed it into the meta-learning algorithms for NIDS. We will investigate new few-shot-based learning frameworks, such as triplet network and contrastive learning methods. Additionally, we will incorporate parallelization mechanisms to further improve the detection efficiency of the method and make it more relevant to practical applications of intrusion detection.

## Figures and Tables

**Figure 1:** The architecture of directed unbalanced few-shot intrusion detection.

**Figure 2:** The distribution of different types of samples in the feature space.

**Figure 3:** Process of unsupervised subtype sampling.

**Figure 4:** Sample spatial distribution of normal traffic after unsupervised subtype sample.

**Figure 5:** The CapsuleNet method.

**Figure 6:** The few-shot capsule network-based NID system.

**Figure 7:** Loss curve.

**Figure 8:** Comparison of detection accuracy of various algorithms: (a) on training A of CICIDS-2017, (b) on training B of CICIDS-2017, (c) on training A of UNSW_NB15, and (d) on training B of UNSW_NB15.

**Figure 9:** Comparison of sampling methods: (a) comparison of optimal sampling results and (b) comparison of multiple experiments.

**Algorithm 1:** Generation of a multiclassification unbalanced few-shot task from the data set.

**Algorithm 2:** Training with DF-Net.

**Table 1:** Compilation of related studies.

Feature	Problem addressed	Method
Network intrusion detection techniques	Machine learning	SVM with feature augmentation [8]
		Improved SMOTE and XGBoost [11]
		Fuzzy analytic hierarchy process and fuzzy TOPSIS [20]
		Multiagent discrete-time Markov decision process (MA-MDP) [21]
	Deep learning	CNN [22]
		Sequential LSTM neural networks autoencoders [6]
		Imbalanced learning and gated recurrent unit neural network [23]
		Spatial-temporal deep neural network [24]
		Combine RNN and CNN [5]
		ANN and autoencoders [25]
		Hierarchical hybrid [26]

Method of unbalanced data processing	Imbalanced data sets	Deep reinforcement learning [27]
		Feature selection and ensemble classifier [28]
		Features dimensionality reduction [29]
		Generative adversarial network [30]
		Adversarial environment reinforcement learning [31]
		CNN based on SMOTE and Gaussian mixture model [14]
		SMOTE [32]
		Variational data generative model [33]
		Modified density peak clustering algorithm and deep belief networks [34]
		Semisupervised *k*-means clustering and posterior probability SVM (PPSVM) [35]

Few-shot learning	Few-shot learning	Prototypical networks [37]
		Relation network [38]
		Matching networks [39]
		Siamese neural networks [40]
	Few-shot learning methods for intrusion detection	Prototypical networks and deep CNN [17]
		Siamese networks and deep CNN [18]

**Table 2:** Experimental data distribution.

Data sets	Definition	Type	Train	Test	Code
CICIDS-2017	Normal	Benign	Sufficient	16,320	iA
	Simulate known attacks	Bot	Sufficient	480	iB
		DDoS	Sufficient	480	iC
		PortScan	Scarce	480	iD
		DoS GoldenEye	Scarce	480	iE
		Web Attack SQL Injection	Scarce	20	iF
	Simulate unknown attacks	DoS Hulk	Zero	1,050	iG
		Heartbleed	Zero	10	iH

UNSW_NB15	Normal	Normal	Sufficient	10,000	rA
	Simulate known attacks	Reconnaissance	Sufficient	600	rB
		Exploits	Sufficient	600	rC
		Analysis	Scarce	600	rD
		Generic	Scarce	600	rE
	Simulate unknown attacks	Backdoor	Zero	583	rF
		Shellcode	Zero	378	rG

**Table 3:** Training set with different sample sizes.

Data sets	Type	Training A	Training B
CICIDS-2017	Benign	27	118
	Bot	11	24
	DDoS	10	19
	PortScan	5	20
	DoS GoldenEye	5	20
	Web Attack SQL Injection	5	10
	Total	63	211

UNSW_NB15	Normal	26	93
	Reconnaissance	15	26
	Exploits	11	31
	Analysis	5	20
	Generic	5	20
	Total	62	190

**Table 4:** Comparison of few-shot intrusion detection methods.

Method	Sample method	*K* value	Algorithm	Loss	Measurement method
FC-NET [18]	Random sampling	Certain	DNN	MSE	Average similarity comparison
Proposed	Unsupervised subtype sampling	Adaptive	CNN + CapsuleNet	Binary cross-entropy	Maximum similarity comparison

**Table 5:** The performance of each method on different evaluation criteria.

Data set	Train set	Method	FP	FN	Accuracy (%)	Precision (%)	Recall (%)
CICIDS-2017	*K* = 5 or training A	FC-NET	1,720	581	88.09	96.16	89.43
		Proposed	**606**	**579**	**93.87**	**96.45**	**96.29**
	*K* = 20 or training B	FC-NET	1,907	510	87.49	96.58	88.31
		Proposed	**587**	**271**	**95.56**	**98.31**	**96.40**

UNSW_NB15	*K* = 5 or training A	FC-NET	1,109	407	88.65	88.91	95.62
		Proposed	**774**	**391**	**91.28**	**92.26**	**95.93**
	*K* = 20 or training B	FC-NET	827	474	90.26	91.73	95.09
		Proposed	**527**	**316**	**93.69**	**94.73**	**96.77**

**Table 6:** Comparison of detection rate (%) of the method to attack type.

Type	*K* = 5 or training A		*K* = 20 or training B	
	FC-NET	Proposed	FC-NET	Proposed
iB	**90.4**	90.0	100.0	100.0
iC	96.3	**96.9**	**100.0**	92.5
iD	65.6	**67.5**	**69.4**	67.5
iE	85.2	**93.1**	94.7	**100.0**
iF	50.0	**55.0**	**95.0**	90.0
iG	**72.0**	70.0	66.3	**93.1**
iH	80.0	80.0	80.0	**90.0**
rB	88.9	**89.0**	91.5	**93.5**
rC	90.7	84.3	89.3	**90.7**
rD	85.1	**86.7**	92.7	87.7
rE	100	97.2	98.2	**99.5**
rF	81.5	**89.5**	74.8	**85.1**
rG	76.2	**80.7**	58.5	**84.9**

**Table 7:** Comparison of detection results of advanced methods.

Data set	Method	Type	Accuracy (%)	Precision (%)	Recall (%)	FLOPs
CICIDS-2017	2018 Flow-based features [58]	CNN + LSTM	97.72	97.97	97.65	70,861
	2020 Random attention capsule [47]	Attention + capsule	98.60	98.59	98.61	31,844
	**Proposed (training A)**	FSL + capsule	95.25	98.37	96.29	94,309
	**Proposed (training B)**	FSL + capsule	96.26	99.07	96.70	

UNSW_NB15	2020 Deep learning-enabled LSTM autoencoder [55]	LSTM + autoencoder	96.0	100	97.0	12,682
	2021 Memory-augmented deep autoencoder [56]	Deep autoencoder	85.30	87.74	85.30	199,004
	2021 Variational LSTM [57]	LSTM	88.30	86.00	97.80	11,219
	**Proposed (training A)**	FSL + capsule	91.28	92.26	95.93	94,309
	**Proposed (training B)**	FSL + capsule	93.69	94.73	96.77	

## Data Availability

We have disclosed the data and source code in our work to facilitate subsequent research and make contribution to the community. The data set used in the article is the public data set CICIDS-2017 and UNSW_NB15 (https://www.unb.ca/cic/datasets/ids-2017.html and https://research.unsw.edu.au/projects/unsw-nb15-dataset).
